The article "High-precision positioning of mine personnel based on wireless pulse technology" was retracted in 2025. Reasons: unreliable results or conclusions; concerns about the peer review.

# High-precision positioning of mine personnel based on wireless pulse technology

**DOI:** 10.1371/journal.pone.0220471

**Published:** 2019-07-31

**Authors:** Xuezhao Zheng, Baoyuan Wang, Ju Zhao

**Affiliations:** 1 School of Safety Science and Engineering, Xi’an University of Science and Technology, Xi’an, China; 2 Key Laboratory of Western Mine and Hazard Prevention, Ministry of Education of China, Xi’an, China; University College London, UNITED KINGDOM

## Abstract

Aiming at addressing current problems of the low accuracy, long delay, and complex arrangement of positioning systems for coal mine workers, a high-precision personnel positioning method based on two round trips of a radio pulse is proposed, and the influencing factors of the positioning by experiments. A matrix is established by taking the transmission timing of the wireless pulse, the preprocessing time of the label, and the receiving time as elements. The result of the matrix calculation shows that the position of the label is related to the above three factors. Experiments are carried out to simulate base station intervals of 20–90 m on an underground roadway. The results show that when the spacing of the positioning base stations is 70 m, the average positioning error is a minimum of 0.0302 m and the positioning delay is a minimum of 0.43 s. In the same experimental environment, after 60 days of continuous operation, it is found that the mean change in the positioning accuracy of the two-round-trip system is within ±0.0003 m while the delay change is within ±0.03 s, showing good system stability.

## Introduction

The main method of coal mining in China is the underground mining of coal seams. The working environment in Chinese coal mines is complex and poor. The situation of coal mine safety in China, in contrast to situations in other developed countries [1], is not optimistic [2]; in particular, five major disasters have accounted for a large proportion of economic losses and casualties in coal mining in China. In recent years, however, Chinese government have gradually increased their emphasis on coal mine safety, constantly improved relevant laws and regulations, strengthened safety supervision, and optimized the production capacity structure of coal mines, thus greatly improving coal mine safety in China and reducing the accident rate [3]. However, coal mining accidents continue to occur in parts of China owing to a large coal output, complicated well mining, and an imbalance of safety and technical support measures. In the period from 2004 to 2015, there were 87 fire-related accidents at coal mines in China, which caused 661 deaths [4–6]. In 2016, China had 197 coal mining accidents, resulting in approximately 451 deaths; the mortality rate per million tons of coal was 0.157, which is much higher than the international standard death rate per million tons of coal (0.02) [7]. The prevention of serious accidents is the most important factor in ensuring the safe operation of coal mines [8]. As an important component of a monitoring system for a coal mine, a personnel positioning system not only monitors the work dynamics of underground personnel in daily production management but also quickly determines the specific location of trapped personnel when disasters occur in coal mines. In the daily management, the geographical location and coordinate information of each staff member can be monitored in detail, and the surrounding environment is roughly divided to ensure that the location of the staff is a mine safety area. In the emergency rescue, the residual positioning node can be used to search for trapped people in the underground, and preliminary detection can be realized according to the area where the pre-disaster personnel are active. It plays an important role in coal mine safety, accident prevention, and emergency rescue [9].

The article "High-precision positioning of mine personnel based on wireless pulse technology" was retracted in 2025. Reasons: unreliable results or conclusions; concerns about the peer review.

China's coal resources are buried deep, and current underground mine roadways and working faces can be 1500 m below the ground [10]. The complicated and variable environment underground and many obstacles interfere with the transmission of electromagnetic waves in the positioning process [11], which reduces the accuracy of personnel positioning. Many scholars have proposed different methods of positioning underground personnel for the safety management of coal mines and the requirements of underground emergency rescue. Awad et al. (2007) proposed a co-localization algorithm on the basis of a distance-based curve component analysis map (CCA-MAP) [12]. The algorithm uses a distance measurement employing received-signal-strength indicator (RSSI) technology. Simulation results show that the algorithm improves positioning accuracy. Fujiwara (2007), Mizugaki et al. (2007), Fujiwara et al. (2008), Halber and Chakravarty (2018) studied a time of arrival (TOA)/time difference of arrival (TDOA) hybrid relative positioning system using ultra-wideband impulse radio (UWB-IR) technology and evaluated the system performance for various distances between base stations through computer simulation and experiment; the positioning error of the system was as low as 22 cm [13–16]. Kim (2009) and Wang et al. (2010) summarized the excitation, principle, and detailed mathematical background of two-way ranging (TWR) and proposed a new ranging algorithm for an asynchronous positioning system, which reduced the number of data packets used in the ranging process and improved the range accuracy [17–18]. Neirynck et al. (2016) proposed an alternative method for the measurement of symmetrical double-sided two-way ranging (SDS-TWR), which eliminated the need for a symmetric recovery constraint. The method effectively uses a timing reference to eliminate clock drift [19]. Peng and Sichitiu (2006) proposed a new angle-of-arrival (AOA) scheme, which can determine direction from a measurement of the angle between adjacent nodes [20]. They showed that even if the measurement is not accurate, there are few beacons and the angle-based method provides better accuracy and precision. Niculescu and Nath (2001) proposed a method by which, assuming that each node has an angle-of-arrival capability [21], only a small number of nodes have positioning capabilities, and all nodes can thus determine their direction and location in an ad-hoc network. Nam et al. (2009) proposed a one-way ranging algorithm based on wireless synchronization with a measurement timestamp and clock frequency offset [22]. The algorithm not only provides instantaneous time information for nodes but also calculates the corresponding distance difference.

The article "High-precision positioning of mine personnel based on wireless pulse technology" was retracted in 2025. Reasons: unreliable results or conclusions; concerns about the peer review.

Comparative analysis reveals that the above methods have large error in positioning and the positioning clock has a large delay [23]. Awad et al (2007) proposed a method that can only achieve a positioning accuracy of 50 cm even in the region of 3.5 x 4.5 m. Although the positioning methods proposed in the literatures has an accuracy of 22 cm, the positioning delay is large and the system layout is more complicated [12–16]. The accuracy of the two-way ranging method depends on the clock drift of the device. The researches show that the improved data transmission can be reduced by improving the ranging algorithm while ensuring the positioning accuracy [17–19]. However, there is no optimization for the time taken for positioning. Other positioning methods have a large delay in locating the clock. The analysis of coal mining practice found three main problems: the first one is time-of-arrival and time-difference-of-arrival positioning methods require that the transmitting device and receiving device clock are accurately synchronized, and the clock frequency offset of the positioning substation and the positioning card in SDS-TWR affects the positioning accuracy, the second one is an underground roadway has a large aspect ratio, and the two-dimensional or three-dimensional positioning error is large and affected by the lack of a line of sight, and the third one is most of the abovementioned ranging positioning methods require high-density node arrangement and additional hardware support, resulting in high energy consumption and a high cost of the positioning system, which are not conducive to the wide-area use of mine positioning.

The article "High-precision positioning of mine personnel based on wireless pulse technology" was retracted in 2025. Reasons: unreliable results or conclusions; concerns about the peer review.

The present paper therefore proposes a positioning technology based on a wireless pulse two-round-trip ranging method of a traditional positioning system. At the same time, owing to the long length and narrow width of the experimental mine roadway [24], the width of the roadway can be neglected in one-dimensional positioning [25]. According to the specific conditions of the experimental roadway, a positioning base station layout network is set up to establish an optimal matching relationship with the positioning label, and the positioning accuracy and delay are optimized and the precision error and delay generated by the system arrangement are minimized.

## Composition of the overall system

Fig 1 shows that the wireless pulse high-precision personnel positioning system mainly comprises reference nodes, gateways, positioning base stations, industrial computers, remote monitoring platforms, and positioning labels worn by underground personnel. The system can be mainly divided into three layers, namely a remote monitoring layer, data transmission conversion layer, and background operation observation layer.

**Fig 1:** Wireless pulse high-precision positioning system.

The remote monitoring layer involves the positioning label, and the transmission of data between a label and positioning base station is carried out by wireless means. The data transmission conversion layer includes the locating of the base stations and converters. The base stations send and receive data packets and record the corresponding times, and converters apply the autonomous localization algorithm to calculate the positioning distance. The background operation observation layer mainly includes an industrial computer and receiver. The client server can change the parameter information of the positioning base station, positioning area, and positioning label, while the web server can play back the track of the positioning label to realize diverse monitoring functions.

### Wireless pulse high-precision personnel positioning technology

#### Working principle and working process of the wireless pulse high-precision positioning system

When miners work on a roadway or at a working face, their positions can be represented by the coordinate movement of their positioning labels. According to the characteristics of wireless communication transmission [26], the maximum layout distance between base stations has been determined to be 100 m. In Fig 2, base stations 1 and 2 are at the centers of circles having different radii between the base station and positioning label.

The article "High-precision positioning of mine personnel based on wireless pulse technology" was retracted in 2025. Reasons: unreliable results or conclusions; concerns about the peer review.

**Fig 2:** Schematic diagram of positioning principle.

The wireless pulse flight time and response flow in the positioning system are shown in Figs 3 and 4. The positioning data packet is sent by any of the positioning base stations, the existing positioning labels and other base stations are identified within the positioning range, and each positioning label pretreats the received data packet immediately and then sends a reply to the positioning base station. To prevent accidental errors resulting from a single measurement, the positioning base station sends the same positioning data packet to the positioning label and other base stations again after receiving the data packet returned by the positioning label. Similarly, the positioning label repeats the last response. After the two positioning responses are completed, the positioning base station takes the average distance between the positioning label and base station 1. Similarly, the distance between the positioning label and base station 2 can be calculated, and the specific position of the label can be determined by combining the two distances.

**Fig 3:** Schematic diagram of the wireless pulse flight time.

**Fig 4:** Two-round-trip positioning flow chart.

#### Distance measurement in wireless pulse positioning

The time calculation of the wireless pulse positioning system mainly includes two measurements of the time taken for the same data round trip between the positioning base station and positioning label. The time taken for a single round trip mainly comprises twice the one-way data transmission time and a label processing time:

$$t_{a1↔t}=\frac{t_{a1}-t_{g}}{2}$$ (1)

$$t_{a1↔t}^{'}=\frac{t_{a1}^{'}-t_{g}^{'}}{2}$$ (2)

where *t*_*ɑ1↔t*_, (ns) is the duration of the first flight of the wireless pulse between base station 1 and the label, *t*_*ɑ1*_, (ns) is the time during which base station 1 sends and receives data packets, *t*_*g*,_ (ns) is the duration of the first pretreatment by the label, *tʹ*_*ɑ1↔t*,_ (ns) is the duration of the second flight of the wireless pulse between base station 1 and the label, *tʹ*_*ɑ1*_, (ns) is the time during which base station 1 sends and receives data packets for a second time, and *tʹ*_*g*_, (ns) is the duration of the second pretreatment by the label. The flight speed of the wireless pulse is multiplied by expressions in Eqs (1) and (2) to give

$$d_{a1↔t}=ct_{a1↔t}=c\frac{t_{a1}-t_{g}}{2}$$ (3)

$$d_{a1↔t}^{'}=ct_{a1↔t}^{'}=c\frac{t_{a1}^{'}-t_{g}^{'}}{2}$$ (4)

$$d_{1}=\frac{d_{a1}+d_{a1}^{'}}{2}$$ (5)

where *c*, is the speed of light, 3 × 10^8^ m/s.

The exact distance between the label and base station 1 can be determined using Eq (5).

The article "High-precision positioning of mine personnel based on wireless pulse technology" was retracted in 2025. Reasons: unreliable results or conclusions; concerns about the peer review.

The time relationship between base stations 1 and 2 and the label is expressed as

$$t_{a1↔a2}+t_{a2}-\Delta T+t_{a1↔a2}^{'}+t_{a2}^{'}-\Delta T^{'}-t_{a1}-t_{a1}^{'}=0$$ (6)

Here *t*_*ɑ1↔ɑ2*_, (ns) is the time during which base station 1 first sends packets to base station 2. This can be obtained from the distance between base stations 1 and 2 ($t_{a_{1}↔a_{2}}=\frac{d_{a_{1}↔a_{2}}}{c}$). *t*_*ɑ2*_, (ns) is the total time during which base station 2 first receives data packets sent by base station 1 and data packets returned by the label. *ΔT*, (ns) is the difference in flight time of packets between base stations 1 and 2 for the first trip. *tʹ*_*ɑ1↔ɑ2*,_ (ns) is the time during which base station 1 sends packets to base station 2 for a second time and is equal to *t*_*ɑ1↔ɑ2*_. *tʹ*_*ɑ2*,_ (ns) is the total time during which base station 2 receives packets sent by base station 1 for the second time and data packets returned by the label. *ΔT'*, (ns) is the difference in the flight time of packets between base stations 1 and 2 for the second trip. The distance between base station 2 and the label can be calculated as

$$d_{a2↔t}=d_{a1↔t}+\Delta Tc$$ (7)

$$d_{a2↔t}^{'}=d_{a1↔t}^{'}+\Delta T^{'}c$$ (8)

Eq (6) can be optimized as

$$t_{a1↔a2}+t_{a2}+t_{a1↔a2}^{'}+t_{a2}^{'}-t_{a1}-t_{a1}^{'}=\Delta T+\Delta T^{'}$$ (9)

Multiplying both sides by the wireless pulse flight speed yields

$$d_{a1↔a2}+d_{a1↔a2}^{'}+c\left[\left(t_{a2}+t_{a2}^{'}\right)-\left(t_{a1}+t_{a1}^{'}\right)\right]=c\left(\Delta T+\Delta T^{'}\right)$$ (10)

In one-dimensional ranging positioning, we take the location of one of the base stations as the origin of coordinates, arrange the two base stations on the axis in the direction of rectangular length, take the direction of rectangular length as the X-axis and the direction of rectangular width as the Y-axis, and establish a local coordinate system. The activity range of the positioning label is always in the plane coordinate system. The distance between the label and base station can be calculated as

$$d=\sqrt{x^{2}+y^{2}}$$ (11)

$$d_{a1↔t}^{2}={\left(x_{a1}-x_{t}\right)}^{2}+{\left(y_{a1}-y_{t}\right)}^{2}$$ (12)

$$d_{a2↔t}^{2}={\left(x_{a2}-x_{t}\right)}^{2}+{\left(y_{a2}-y_{t}\right)}^{2}$$ (13)

where *d*_*ɑ1↔t*,_ and *d*_*ɑ2↔t*_, are the distances between the label and base stations 1 and 2 while (*x*_*t*_,*y*_*t*_)denotes the actual coordinates of labels. Subtracting the expression in Eq (12) from the expression in Eq (13) yields

$$d_{a2↔t}^{2}-d_{a1↔t}^{2}=x_{a2}^{2}-x_{a1}^{2}-2x_{a2}x_{t}+2x_{a1}x_{t}+y_{a2}^{2}-y_{a1}^{2}-2y_{a2}y_{t}+2y_{a1}y_{t}$$ (14)

$$2\left[\left(x_{a1}-x_{a2}\right)x_{t}+\left(y_{a1}-y_{a2}\right)y_{t}\right]=d_{a2↔t}^{2}-d_{a1↔t}^{2}+x_{a1}^{2}-x_{a2}^{2}+y_{a1}^{2}-y_{a2}^{2}$$ (15)

$$2\left[x_{a1}-x_{a2}\;y_{a1}-y_{a2}\right]\left[\begin{array}{l} x_{t}\\ y_{t} \end{array}\right]=[d_{a2↔t}^{2}-d_{a1↔t}^{2}+x_{a1}^{2}-x_{a2}^{2}+y_{a1}^{2}-y_{a2}^{2}]$$ (16)

Squaring both sides of Eq (7) yields

$$d_{a2↔t}^{2}=d_{a1↔t}^{2}+2d_{a1↔t}\Delta Tc+\Delta T^{2}c^{2}$$ (17)

$$d_{a2↔t}^{2}-d_{a1↔t}^{2}=2d_{a1↔t}\Delta Tc+\Delta T^{2}c^{2}$$ (18)

$$d_{a2↔t}^{2}-d_{a1↔t}^{2}=c\left(t_{a1}-t_{g}\right)\Delta Tc+\Delta T^{2}c^{2}$$ (19)

Substituting Eq (19) into Eq (16) yields

$$2\left(x_{a1}-x_{a2}\;y_{a1}-y_{a2}\right)\left[\begin{array}{c} x_{t}\\ y_{t} \end{array}\right]=\left[c\left(t_{a_{1}}-t_{g}\right)\Delta Tc+\Delta T^{2}c^{2}+x_{a1}^{2}-x_{a2}^{2}+y_{a1}^{2}-y_{a2}^{2}\right]$$ (20)

Eq (20) shows that the specific location of the positioning label can be identified by combining *t*_*ɑ1*_,*t*_*g*_, *ΔT*, (*x*_*ɑ*1_, *x*_*ɑ2*_, *y*_*ɑ1*_, *y*_*ɑ2*_)as known coordinate information) without the effect of the clock offset frequency.

The article "High-precision positioning of mine personnel based on wireless pulse technology" was retracted in 2025. Reasons: unreliable results or conclusions; concerns about the peer review.

## Field test and analysis

### Precision verification experiment

The base station separation distance is selected to range from 20 to 90 m to ensure the effectiveness of the base station arrangement and the reliability of the wireless transmission. Different sets of eight experiments are performed separately. The experimental site is chosen to simulate a roadway underground. The roadway has a length of 90 m and width of 4 m and is rectangular with an aspect ratio close to 23:1. This selection is more in line with the one-dimensional ranging principle performed by the above algorithm, and there is no label drift phenomenon. Using the principle of the control variable method, under the premise of ensuring that the distance between the base stations is constant, the position of the label is constantly changed, and the position coordinates of the positioning label can be obtained on the background server. Because the base station is not the primary slave, the positioning accuracy between two base stations can be studied only by analyzing the positioning error within half the distance between them. The distance between the base station at the origin of coordinates and the midpoint of the two base stations is denoted *z*. The base station is taken as the starting point, and the positioning accuracy of labels is measured between 0.1*z* and *z*.

Criteria commonly used to evaluate the accuracy of positioning algorithms include the root mean square error, mean square error, geometric precision factor, Cramer–Luo lower bound, and cumulative distribution function. This paper experimentally determines the coordinates of the positioning label and therefore uses the root mean square error to evaluate the positioning accuracy [27]. To clearly reflect the size and trend of the positioning error for different base stations, it is defined that

$$\varepsilon_{RMSE}=\sqrt{\frac{1}{N}\overset{N}{\underset{i=1}{\sum }}\left[\left({\hat{x}}_{l}-x_{i}\right)2+\left({\hat{y}}_{l}-y_{i}\right)\right]}$$ (21)

where *N* is the number of measurements and (${\hat{x}}_{l},{\hat{y}}_{l}$) is the observed value of the positioning label on the background server. To reduce accidental error due to individual differences of the labels, three different labels are placed at the same position. The average value of the three positioning accuracy errors is used as the final error:

$$\varepsilon_{RMSE}=\left(\varepsilon_{RMSE1}+\varepsilon_{RMSE2}+\varepsilon_{RMSE3}\right)÷3$$ (22)

where *ε*_*RMSE1*,_ *ε*_*RMSE2*,_ *ε*_*RMSE3*_ represent the different positioning accuracy errors of the three labels. The distance between base stations is respectively set as 20, 30, 40, 50, 60, 70, 80, and 90 m in what are referred to as experiments 2, 3, 4, 5, 6, 7, 8, and 9. Results are presented in Figs 5–13. To reflect the size and trend of positioning error for different base stations clearly, we define

$$\phi =\varepsilon_{RMSE}\times 100\%$$ (23)

δ=1−ϕ (24)

where *∅*, is the error coefficient and *δ*, is the exact coefficient.

The article "High-precision positioning of mine personnel based on wireless pulse technology" was retracted in 2025. Reasons: unreliable results or conclusions; concerns about the peer review.

**Fig 5:** Error in experiments 2–9.

**Fig 6:** Error in experiment 2.

**Fig 7:** Error in experiment 3.

**Fig 8:** Error in experiment 4.

**Fig 9:** Error in experiment 5.

**Fig 10:** Error in experiment 6.

**Fig 11:** Error in experiment 7.

**Fig 12:** Error in experiment 8.

**Fig 13:** Error in experiment 9.

Fig 5 shows that the positioning accuracy error is less than 2 m for separations of the base stations of 20–90 m. However, when the distance between base stations is 90 m, the error differs greatly at different positions, the positioning error is mostly greater than 0.4 m and the maximum error exceeds 1.5 m, and some accuracy coefficients are negative. This distance is therefore not considered appropriate. Figs 6–13 present the relation between the precision error coefficient and accuracy coefficient for different base station separations. For all separations, the positioning error coefficient of the system is less than 20% and changes little. When the distance between base stations is 20–70 m, the positioning error coefficient is less than 15%. High-precision positioning means that more than 95% comprehensive ranging positioning error does not exceed ±1 m, which meets the requirement of high accuracy [28].

### Positioning delay test

In order to verify the delay of the positioning system, based on the test conditions of the positioning accuracy experiment, the delay of the positioning tag when measuring the distance between the base stations is measured. The average of delays for three labels is taken as the delay of the positioning label. To simplify the model of the positioning label delay test, this experiment takes the time that the label reaches the base station as the test time, and the tester moves forward between the positioning base stations at a normal walking speed. It is ensured that the position of the positioning label is stable before starting the test. As the tester begins walking, the tester and background observer simultaneously record the time. When the tester arrives at the horizontal line of the base station, the tester records the actual time of arrival. At this time, the label seen by the delayed background observation has not passed the horizontal line of the base station. A diagram of the experiment is shown in Fig 14. The average time delay of the system *Δt*_*sum*_ (s) is

**Fig 14:** Schematic diagram of the positioning delay.

$$\Delta t_{sum}=\frac{\sum_{i=1}^{3}\left[\left(t_{ri}-t_{si}\right)-\left(t_{ai}-t_{si}\right)\right]}{3}$$ (25)

where *t*_*s*,_ (s) is the start time, *t*_*ɑ*,_ (s) is the actual arrival time, and *t*_*r*,_ (s) is the time that the background observation reaches the specified position. Test results are presented in Table 1 and Fig 15.

The article "High-precision positioning of mine personnel based on wireless pulse technology" was retracted in 2025. Reasons: unreliable results or conclusions; concerns about the peer review.

**Fig 15:** Curve of location delay time and base station distance.

**Table 1:** Base station distances and system delays.

Distance between base stations/m	20	30	40	50	60	70	80
**System delay/s**	1.72	0.88	1.24	0.5	0.49	0.43	1.39

Table 1 shows that the system delay ranges from 0.43 s (for a separation of base stations of 70 m) to 1.72 s (for a separation of base stations of 20 m) as the separation of base stations ranges 20–80 m. This is because the required flight time is short and the system delay time improves when the base stations are close. The flight time of the wireless pulse increases with the distance between the base stations, which worsens the system delay. However, the flight distance of the wireless pulse increases as the distance between the base stations increases, causing the system delay time to increase again. Fig 15 reveals that the positioning delay time is within 0.5 s when the distance between base stations is 50–70 m, which meets the requirement of a small delay [29]. According to reference 29, the signal delay is less than half of the signal duration, which is a low delay. In this paper, the duration of the signal can be regarded as the difference between the maximum delay time and the minimum delay time of the system, and the duration of the system is 0.645s.

The article "High-precision positioning of mine personnel based on wireless pulse technology" was retracted in 2025. Reasons: unreliable results or conclusions; concerns about the peer review.

### Experiment on the optimization of the base station layout

For the same experimental environment and base station arrangement as in the positioning accuracy experiment, the positioning error was analyzed for different separations of the base stations in the range of 20–80 m. Test results are presented in Tables 2 and 3 and Figs 16 and 17.

**Fig 16:** Errors in different test distances for separations of positioning base stations ranging 20~80 m.

**Fig 17:** Comparison of three errors separations of positioning base stations ranging 20~80 m.

**Table 2:** Positioning accuracy for different label positions and base station separations.

	Multiples from the Midpoint of the Base Station	0.1	0.2	0.3	0.4	0.5	0.6	0.7	0.8	0.9	1
**Distance between Base Stations/m**	**20**	0.105	0.131	0.140	0.075	0.009	0.034	0.001	0.009	0.047	0.008
	**30**	0.016	0.095	0.033	0.019	0.001	0.063	0.034	0.016	0.026	0.079
	**40**	0.029	0.092	0.037	0.007	0.011	0.049	0.082	0.061	0.052	0.094
	**50**	0.071	0.015	0.071	0.039	0.047	0.066	0.018	0.074	0.091	0.036
	**60**	0.107	0.107	0.102	0.107	0.078	0.063	0.080	0.032	0.087	0.004
	**70**	0.149	0.024	0.003	0.021	0.014	0.004	0.040	0.019	0.023	0.005
	**80**	0.165	0.203	0.086	0.027	0.014	0.204	0.064	0.171	0.023	0.005

**Table 3:** Three error values for different base station separations.

Distance /m	20	30	40	50	60	70	80
**Maximum /m**	0.140	0.095	0.094	0.091	0.107	0.149	0.171
**Average value /m**	0.0559	0.0382	0.0514	0.0528	0.0767	0.0302	0.0962
**Minimum /m**	0.001	0.001	0.007	0.015	0.004	0.004	0.005

Fig 16 reveals that when the distance between the base stations is 20–80 m, the positioning error of the label is less than 0.2 m at different test distances from the midpoint of the base stations. The error of the positioning label at different distances from the base station is a minimum when the separation of base stations is 70 m. It is determined that the distance between base stations is 70 m, which is the optimal arrangement separation of base stations for the positioning method. Fig 17 reveals that the maximum positioning error is less than 0.18 m, the average value is less than 0.1 m, and the minimum value is close to zero when the base station separation is 20–80 m; i.e., three different positioning errors can be used as the standard of the positioning system accuracy.

### System runtime test

Taking into account the limitations of coal mine working hours and system power supply issues,to verify the effect of the system running continuously in a coal mine, an experiment was carried out on precision and delay over 60 days at intervals of 5 days for the optimal separation of base stations of 70 m. Two methods were used to judge whether the accuracy worsens or the delay increases. Results are presented in Tables 4 and 5 and Figs 18 and 19.

The article "High-precision positioning of mine personnel based on wireless pulse technology" was retracted in 2025. Reasons: unreliable results or conclusions; concerns about the peer review.

**Fig 18:** Changes in positioning accuracy for a separation of positioning base stations of 70 m on different days.

**Fig 19:** Positioning delay variation for a separation of positioning base stations of 70 m on different days.

**Table 4:** Change in positioning accuracy over time.

Day/d	5	10	15	20	25	30	35	40	45	50	55	60
**Precision/m**	0.0301	0.0299	0.0302	0.0303	0.0305	0.0301	0.0302	0.0303	0.0302	0.0301	0.0304	0.0302
**Average Accuracy/m**	0.0302	0.0302	0.0302	0.0302	0.0302	0.0302	0.0302	0.0302	0.0302	0.0302	0.0302	0.0302
**Error/m**	-0.0001	0.0003	0	0.0001	0.0003	-0.0001	0	0.0001	0	-0.0001	0.0002	0

**Table 5:** Positional delay change on different days for a base station separation of 70 m.

Day/d	5	10	15	20	25	30	35	40	45	50	55	60
**Delay /s**	0.41	0.42	0.44	0.40	0.45	0.42	0.47	0.44	0.42	0.45	0.46	0.43
**Average delay/s**	0.43	0.43	0.43	0.43	0.43	0.43	0.43	0.43	0.43	0.43	0.43	0.43
**Error/s**	-0.02	-0.01	0.01	-0.03	0.02	-0.01	0.04	0.01	-0.01	0.02	0.03	0

Tables 4 and 5 show that the positioning accuracy of the system remains high with time; the accuracy does not fall by more than ±0.0003 m and the average change in accuracy over time is 0.00026 m. It is thus considered that the accuracy does not change. The change in the positioning delay is small, the delay variation remains within 0.03 s, and the average delay variation over 60 days is 0.0175 s. It is thus considered that the positioning delay does not change. As can be seen in conjunction with Figs 18 and 19, fluctuations of the positioning accuracy and positioning delay are small in the experimental period, and both the accuracy and delay fluctuate above and below zero, so that the positioning system does not have a large offset during its running time.

In order to analyze the application effect of various positioning methods in coal mines, the positioning accuracy and positioning delay are compared with this method. The specific results are shown in Table 6.

**Table 6:** Comparison between TOTF positioning methods and other underground mine personnel positioning methods.

	Comparison parameter	Positioning accuracy	Positioning delay	Mine suitability
**Positioning methods**	**RSSI**	Low (>50cm)	Higher (>2s)	Poor
	**TOA**	Lower (>22cm)	Higher (>2s)	Worse
	**AOA**	Low (>50cm)	General (>1.5s)	Poor
	**TDOA**	General (>20cm)	Lower (>1s)	General
	**TWR**	Higher(>15cm)	Low (>1s)	Better
	**SDS-TWR**	High (>10cm)	Lower (>1s)	Well
	**The method(TOTF)**	High (10cm)	Low (>1s)	Well

In the normal production process of underground coal mines, personnel positioning is affected by the structure of the roadway, the distribution of obstacles, the distance between substations and the frequency of clock drift. Therefore, positioning accuracy, positioning delay and the applicability of positioning method are needed to consider synthetically. The positioning in the paper only needs to arrange the distance between the substations reasonably, and has no relationship with the signal strength, the transmission and reception time caused by the clock drift. The positioning accuracy is not affected by the signal transmission power, the receiving sensitivity and the transmission attenuation caused by other obstacles; the positioning delay is also independent of personnel density, staff distribution, and location tag synchronization. In particular, the method does not distinguish between the master and slave base stations, greatly reduces the complexity and delay between the systems, and has good applicability to complex buildings like mine. Based on the above analysis, the application results of RSSI, TOA and AOA in coal mines are poor. TDOA, TWR and SDS-TWR have good application effects, and are currently widely used in coal mines. This method is better than other methods. The positioning method has great advantages in both positioning accuracy and positioning delay. Therefore, it can be predicted that the method has great research and secondary development significance in the future.

The article "High-precision positioning of mine personnel based on wireless pulse technology" was retracted in 2025. Reasons: unreliable results or conclusions; concerns about the peer review.

## Conclusion

Aiming at the problems of a high precision error and obvious delay in the positioning of mine personnel, this paper conducted relevant theoretical research and developed an algorithm for high-precision personnel positioning using a wireless pulse. An underground experiment was conducted. The study made the following contributions.

1. The architecture of a positioning system based on wireless pulse two-round-trip flight time ranging was proposed, and a prototype was developed. Experimental results show that the system meets actual requirements.
2. A one-dimensional ranging location algorithm was proposed and optimized according to the flight time of the wireless pulse, label preprocessing time, and recorded time correlation matrix of the base station.
3. Experimental results show that the optimal spacing of base stations on a mine roadway is 70 m; the error coefficient is less than 15%, the error average is 0.0302 m, and the positioning delay is less than 0.5 s. In addition, continuous testing over 60 d of system running time found no appreciable change in the precision or delay.
4. The TOTF positioning method is superior to other existing mine positioning methods in terms of positioning accuracy, positioning delay, and applicability to coal mines.
